The article "Healthcare Facilities Redesign Using Multicriteria Decision-Making: Fuzzy TOPSIS and Graph Heuristic Theories" was published in 2023. Journal: J Healthc Eng.

# Healthcare Facilities Redesign Using Multicriteria Decision-Making: Fuzzy TOPSIS and Graph Heuristic Theories

**DOI:** 10.1155/2023/9648510

**Published:** 2023-02-16

**Authors:** Amr A. Hassanain, Mohamed A. A. Eldosoky, Ahmed M. Soliman

**Affiliations:** ^1^Biomedical Engineering Department, Faculty of Engineering, Helwan University, Cairo 11795, Egypt; ^2^Faculty of Engineering, Egyptian Chinese University, Cairo, Egypt

## Abstract

**Background:**

Healthcare facilities are crucial assets that are necessary to be updated and evaluated regularly. One of the most pressing issues today is the renovation of healthcare facilities to match international standards. In large projects involving nations renovating healthcare facilities, it is necessary to rank the evaluated hospitals and medical centers in making optimal decisions for the redesign process.

**Objective:**

This study presents the process of renovating old healthcare facilities to meet international standards, applying proposed algorithms for measuring compliance for redesign, and deciding whether or not the redesign process is beneficial.

**Methods:**

The evaluated hospitals were ranked using a fuzzy technique for order of preference by similarity to ideal solution algorithm and a reallocation algorithm that calculates the layout score before and after applying the proposed algorithm for the redesign process using bubble plan and graph heuristics techniques. *Results and Conclusion*. The results of the methodologies applied to 10 evaluated hospitals as selected hospitals in Egypt showed that the hospital with the abbreviation (D) had the most required general hospital criteria, and the hospital with the abbreviation (I) had no cardiac catheterization laboratory and lacked the most international standard criteria. After applying the reallocation algorithm, one hospital's operating theater layout score improved by 32.5%. Proposed algorithms support decision-making by helping organizations redesign healthcare facilities.

## 1. Introduction

Ranking a hospital means dealing with a vast amount of data. By comparing several aspects of quality and service, rankings are typically achieved. Evaluating a hospital's standard patient healthcare is multidimensional: it involves comprehensive patient-care experiences. Indicators of hospital performance are now used to evaluate and compare hospital performances. To achieve these goals, hospitals should be ranked according to the quality of their care based on quality indices. Initiating quality assurance measures is based on these evaluations, which have become progressively crucial in recent years [1]. As a result, the public's interest in hospital rankings has grown in recent years [2]. Accurate hospital performance evaluations are essential in this context. Hospitals may vary when assessing risk variables, such as the demographic structure or illnesses in a patient. Quality indicators are generally thought of as risk-adjusted to address this issue.

Healthcare systems have improved in rural and remote areas over the past few decades, but a new reality is on the horizon. It is becoming more and more difficult for health systems to generate better outcomes and higher societal value because of changing medical needs, increased public expectations, and new health objectives. However, continuing the current course will fall short of meeting these needs. What is required are elevated healthcare systems that continuously deliver healthcare that either improves or maintains good health by being respected and trusted by all individuals and by reacting to changes in demographic demands. Quality should not be a luxury for a select few or an idea long-term; it should be ingrained in all health systems. Human health rights are useless without high-quality healthcare, which is impossible without a functioning healthcare system that can provide it.

Converging various economic and social aspects, healthcare systems now strive to give the greatest services at the lowest cost, seeking maximum efficiency and efficacy. Hospitals are among the most complicated building types because of their diversified and numerous daily users, the huge integrated technology and systems, and the structure's role as an open arena for improving the public's health and well-being. When constructing and expanding healthcare facilities, it is common for these facilities to be developed and expanded over decades. Medical facilities are necessary to be adaptable to the impending 80% shift in medical and technological knowledge in the next two decades [3]. The future of healthcare is fraught with peril given that 40% of hospitals today do not follow the modern functional and technical paradigm (pavilion design and low ceiling). Due to the hospital's age and accelerating obsolescence trend, the existing health culture cannot meet the needs of such modifications in the contemporary setting.

Health systems should be rated largely on their health outcomes, such as greater health and more fair distribution, the trust people have in their health system, and their economic gain, including competent service and positive user experiences. Population and health needs and requirements, governance of the health sector, and cross-sectoral collaborations and channels for care delivery are some of the pillars of high-quality health systems. In addition to having solid foundations, health systems are necessary to evaluate and use data to learn. People should be the focus of health systems, and they should be equal and resilient as well as productive.

Hospitals in the 21st century should be organized and funded to encourage all kinds of healthcare exchanges that promote information transfer and enhance the curing connection [4].

Even in the digital age, clinician-patient interaction is still a vital part of many people's healing; face-to-face encounters are essential. Clinical examination and observation of the patient's demeanor are also possible during face-to-face appointments. However, face-to-face interactions are neither desired nor necessary by both the therapist and the patient in many circumstances. Using electronic communication instead of face-to-face encounters can improve efficiency and achieve the best possible outcomes.

It may also be useful to free up more clinician time for face-to-face visits by judiciously using electronic and other modes of communication. As a result of the current healthcare system, face-to-face encounters are routinely rushed or deferred. During the appointment, there may not be enough time to fully explore the underlying psychological causes of symptoms or how they are linked to other underlying health issues. Moreover, there may not be enough time to educate the patient and family members about a medical condition and provide enough supportive care for the pain, despair, and loss accompanying the sickness [5].

The study solved problems that exist in hospitals, in general, using redesign algorithms to help decision makers for optimal solutions and improving the current status of the healthcare facilities as discussed in the methodology and result sections.

## 2. Literature Review

### 2.1. Assess the Need for a Significant Redesign

First, the leadership must determine whether the organization can embark on a substantial redesign or system transformation. Identifying and analyzing previous redesign attempts is critical for both the management and the people. Those responsible for administering the projects should create a document that describes project goals, identifies whether or not they were accomplished, describes the impediments to attaining the goals, outlines the variables that contributed to the success, and identifies knowledge gained.

People will feel more confident about tackling a system redesign when they see earlier projects and know the company has performed it before. Examples include Denver Health's recent initiatives to improve business and clinical operations. Changes to the business model included the handover of the entire system to an autonomous government agency. A comprehensive information technology strategy for the entire hospital should be implemented. All aspects of behavioral health have been restructured and integrated with other systems and primary care processes, and an open access system has been implemented—a well-planned community outreach campaign.

### 2.2. Establish the Redesign Perspectives

To understand the redesign process clearly, several points of view should be considered. With these viewpoints in mind, efforts are better directed to process improvement. To successfully restructure healthcare systems, numerous concurrent viewpoints appear beneficial and required. Quality, safety, customer care, productivity, infrastructure environment, and employment services, including doctor development, should be included in the concepts for redesign and relevant activities for system-wide innovation.

Transformation can be driven from various viewpoints, including architecture, quality, service quality, employee development, quality care, and efficiency. For example, focusing on quality can lead to processes that benefit both the product and the consumer. The company's culture embraces and fosters a diversity of viewpoints. Information technology plays a key role in facilitating these process changes. Instead of being the catalyst for change, information technology serves as a means to that end. An important redesign initiative in Sweden's Jonkoping County Council was called “The Esther Project,” giving it a human face and emphasizing the importance of rethinking healthcare delivery from general care to medical care [6].

### 2.3. Organize the Redesign Process into a System

Architecture for redesign requires three components: a point person to manage the process, a team to oversee the planning method, and a broad-based corporate group of leaders and cheerleaders to support the project. The more senior the individual leading the redesign effort, the more likely it is to be implemented and perpetuated. As long as a senior hospital official leads the initiative, all personnel will value it. In addition, a core team must be established. This group is responsible for implementing many of the simple methods in use. This varies greatly on the project's scope. In any case, one individual must take on the project manager position and know the magnitude of the project. Those who can gather, analyze, and interpret data must be part of the core team. It is critical to have an industrial or operations management engineer on the project team.

### 2.4. Gather External Information

Both healthcare and nonhealthcare reform literature should be reviewed. In the event of a site visit, one must determine where to go, whom to send, and what information to collect. According to this recommendation, site visits or conference calls should involve representatives from the healthcare and nonhealthcare sectors. Nonhealthcare industries have a lot to offer, and they must be included.

Healthcare systems have not yet attained the same level of innovation as other industries, but it is still worthwhile to visit them. As a result of these industries' efforts, quality, productivity, customer support, and safety have improved. In the healthcare setting, some of these methods and concepts can be used to rethink healthcare systems [7].

There should be a clinician, an analyst, and a director of the Internal Working Group on the team, including a clinical person. All team members should attend site visits and conference calls. Additionally, these visits help to cultivate leaders within the organization. The studies that apply some ranking methods will be discussed as shown in Table 1, and the benefits and limitations of TOPSIS (technique for order of preference by similarity to ideal solution), MOORA (multiobjective optimization on the basis of ratio analysis), VIKOR (VlseKriterijumska Optimizacija) (multicriteria optimization and compromise solution), PROMETHEE (preference ranking for organization method for enrichment evaluation), and SAW (simple additive weighting) methods will be discussed as shown in Table 2.

There are new methods used in the ranking, such as COMET (Characteristic Objects Method), which enables relatively easy identification of both linear and nonlinear expert decision functions; use of global criterion weights, which determine the average significance of a given criterion for the final assessment; and helps a DM (decision-maker) to organize the structure of the problems to be solved and carry out the analysis, comparisons, and ranking of the alternatives, completely independent of their number. The proposed approach enables the identification of the whole domain model, is resistant to the rank reversal phenomenon, is easy to apply, and allows the generation of an objective and reliable recommendation based on the gathered data. It is far superior to the TOPSIS or AHP methods [29, 30].

The method V-COMET (V-Characteristic Objects Method) is characterized by high accuracy and has very limited computational complexity. It delivers two solutions to the same problem using the same data but two different procedures; because both solutions normally coincide, this agreement provides a high level of reliability. The model not only delivers solutions but also informs on aspects that are related to the selection achieved. The method mixes human knowledge, expertise, and know-how with a scientific approach, giving the decision-maker a solid foundation for his/her final decision [24, 28].

The method CODAS-COMET eliminates the limitations of COMET by automatizing and accelerating the characteristic object comparison procedure [31].

## 3. Methodology

### 3.1. Research Design

The research talks about the ranking of evaluated hospitals and the redesign process of existing hospitals, if applicable. The choice of the facilities to take part in the study will be identified. The goal is to further develop methods that aid in making appropriate decisions for health facilities, guaranteeing that their structures are in accordance with internationally accepted standards and ensuring high-quality performance across the hospitals by helping a mobile-based application with intelligent (HFBEE) in the evaluation process. Due to the nature of the study, it will be quantitative. A quantitative study is referred to as a systematic approach meant to investigate a particular phenomenon [33], and the result is to derive a technique to rank an appropriate decision-making redesign process for evaluated hospitals.

### 3.2. Target Population

The research intends to target health facilities across the Middle East to create a healthy working environment. Health facilities should create the right standards during their operations, accrediting international or local governing principles. It means creating an environment where all respective operations are working in strict adherence to the generally accepted ways of conduct and ensuring the safety of all stakeholders. Hospitals remain one of the most important institutions in the Middle East; they operate under the ministers of health, ensuring that the health of individuals is preserved by guaranteeing adequate healthcare and, most importantly, creating a conducive operating environment for all health institutions.

### 3.3. Sample Size and Selection

The research intends to have a significant number of samples for the study. Sampling will ensure the predetermination of various research variables from the participants [34]. Therefore, a substantial number of participants will assist in observing distinct characteristics that will assist in creating an appropriate algorithm to be used in the mobile-based application for evaluating and weighing the hospitals. The study will adopt a randomized sampling procedure. It will allow various health facilities to participate in the study based on the random sampling procedure, where every institution carries equal chances of participating in the study.

### 3.4. Study Area

The study will take place in upper Egypt. Over the years, the region has witnessed significant developments in the health sector attributed to the massive developments and demand in the health sector. Health facilities are equally emerging across the city due to the growing healthcare pressure. Due to the massive growth of the health sector in Egypt, a few studies exist expounding on the need to rank and weigh these hospitals. The typical aim of ranking and weighting ensures that healthcare institutions arrive at various policy goals. It is also understandable that, due to the growing pressure, decision-making in healthcare is quite complex and basically surrounded by a range of conflicting aims.

### 3.5. Data Collection Procedure

Data collection involve a systematic procedure where various observations and measurements are equally provided. The main purpose of this research is to rank the evaluation of hospital departments in Egyptian healthcare facilities. As a result, the researcher uses an Android software application as a questionnaire to be administered to healthcare institutions. The goal is to find out the application of the ranking methods in the specific evaluated healthcare facilities. Furthermore, the purpose of the proposed algorithms is to elaborate on the problems faced by Egyptian health facilities in their decision-making activities. When enough evidence is gathered, it will be feasible to introduce an application assisting these health facilities during their decision-making activities.

### 3.6. Data Analysis and Presentation

Data analysis will follow after data collection and is satisfied. The purpose is to ensure the raw data are cleaned, transformed, and modeled to discover useful patterns [35]. These findings will be then presented using computational techniques and, finally, developing a proper algorithm to solve decision-making complexities found in Egyptian health facilities.

### 3.7. Development of Algorithm Models

Based on the ranking and weighting standards, it is important to develop an algorithm to be used in decision-making. The optimal aim of the study is to ensure that health facilities are assessed in terms of their capabilities to offer design standards. Most healthcare organizations face critical challenges when it comes to making decisions, and it is for this purpose that makes it difficult to get accurate undertakings about their operations. The algorithms herein present an overview of our approach toward the ranking and reallocation of hospital departments for proper decisions.

#### 3.7.1. Ranking Algorithm

*(1) Fuzzy Sets*. Honesty, optimism, and/or mental measurements are not precise and absolute. “How is your health? How is your income?”

The answers to these questions are neither precise nor clear (nonmetric) but more such as “well” and “very well” and therefore in the “moderate” form. These answers have in common that they are fuzzed. They are not clear like black or white but are expressed in gray. Answers containing uncertainty (or being gray) should be considered throughout our daily lives as we often come across them. The expression of Andre Gide, “colour of truth is gray,” highlights the importance of the uncertainty feature in our everyday lives. Linguistic variables are words in which values contain uncertainty or fuzziness. If the decision-making problem procedure used linguistic variables for which values have imprecise categories, it is obvious that the results would be closer to the truth. In this paper, we state fuzzy sets as shown in Figure 1 [36] and their linguistic scale as shown in Table 3.

Fuzzy set boundaries are a noncollection of crisp elements, so staff members in the transition to becoming nonmembers are gradual, not sudden. The rule of fuzzy set theory is that an element can be joined partially to the fuzzy set. A set of *x* elements gets *X*. Let *A* be defined as a fuzzy set. If *A* (*x*) = 1, then *x* completely belongs to the set of *A*. If *μA* (*x*) = 0, then *x* does not belong to *A*. For this reason, 0 > *A* (*x*) > 1, *x* partially belongs to

(1) $$\begin{array}{c} \mu_{c}\left(x\right)=\left\{\begin{array}{c} \begin{array}{cc} \frac{\left(x-k\right)}{\left(l-k\right)}\text{,} & for\;k\leq x\leq l \end{array}\text{,}\\ \begin{array}{cc} \frac{\left(x-m\right)}{\left(l-m\right)}\text{,} & for\;l\leq x\leq m, \end{array}\\ \begin{array}{cc} 0\text{,} & other\;wise \end{array}\text{.} \end{array}\right) \end{array}$$

Triangular membership functions are often used because of the convenience of calculation.

The parameters *k* and *m*, respectively, set the lower and upper limits of the fuzzy number; the *l* parameter determines the center of the fuzzy number, the membership function of where *A* (*x*) = 1 is represented by the *C*. *l* parameter. As a result, fuzzy number *C* = (*k*, *l*, *m*) indicates a fuzzy value “approximately l.” This value cannot be smaller than *k* or bigger than *m*. The membership value increases linearly from *k* to *l* and decreases from *l* to *m*. Variables whose values are qualitative words in natural languages are called linguistic variables [37]. Linguistic variable values are not numbers; they are rather words or sentences of natural or artificial language [38]. A linguistic variable *Q* consists of terms, so in fact, linguistic values of *Q* are fuzzy sets. Figure 1 shows triangular membership functions of linguistic values as not all satisfied, can be satisfied, and not applicable.

The reason for using triangular fuzzy numbers is that they can easily be expressed for decision-makers.

As identified through the literature, healthcare decisions remain quite a challenge. This is attributed to the multiple trade-offs among conflicting goals and objectives. However, structured decision-making activities create relative models meant to solve these occurrences. For this part, the most suitable algorithm is the technique for order of preference by similarity to ideal solution (TOPSIS). Its purpose is to ensure that appropriate ranks are granted to the hospital's strategies toward improving its service delivery per Egyptian and other international hospital standards. The ranking algorithm 1 is to assist in the formulation of accurate decisions, as shown in Figure 2.

#### 3.7.2. Reallocation of Department's Area Algorithm

Algorithm 2 prepared for improvement the facility layout, which can arrange the department's spaces as possible to enhance the present layout [38].

#### 3.7.3. Decision-Making Algorithm

The evaluation, ranking, and reallocation of the department's area algorithm will critically allow the redesign of these health facilities, prompting them to fit into current requirements and update their operations. These will, in turn, lead to accurate decisions and the gathering of accurate information regarding the operations, as shown in Figure 3.

### 3.8. Case Study: Sample and Setting

A hospital's evaluation composed of 1458 questions was divided into 13 departments derived from seven international standards guidelines and accreditation programs for 10 public hospitals in Egypt. The hospital (unidentified for legal reasons) is in the upper of the country. The hospital integrates a local health unit, resulting from a vertical merging of one hospital and several nearby primary health centers. The characteristics *s* of the selected hospitals are shown in Table 4. The evaluation is carried out using Android software (HFBEE) and ranking the departments of the selected 10 hospitals using the proposed algorithm. The evaluation proceeded using the international standards of healthcare facilities design as shown in Table 5, and these standards criteria were weighted using entropy technique [38]. The proposed algorithm 2 is applied to one selected hospital to test and validate the redesign decision-making algorithm.

## 4. Results and Discussion

In this research, the selected evaluated hospitals as a case study after the analysis appeared to make clear decisions for the redesign or renovation process. The selected evaluated hospitals' ranking results of their departments are shown in Table 6.

### 4.1. Operating Theatre Reallocation Case Study

The reallocation process of the high compliance departments showed that the layout score before applying the proposed algorithm for reallocation is 28%. The operating theater at hospital F is shown in Figure 4.

**Step 1 .**

extracted adjacency matrix from the proposed adjacency matrix as shown in Table 7 for the operating theater department in hospital F.

**Step 2 .**

extracted REL chart as shown in Table 8 for the operating theater department in hospital F.

Using

(2) $$\begin{array}{c} {LS}^{a}=\overset{M-1}{\underset{i=1}{\sum }}\overset{M}{\underset{j=j+1}{\sum }}V\left(r_{ij}\right).a_{ij}\text{.} \end{array}$$

Layout score = 28.

**Step 3 .**

adjacency matrix for the operating theater department as optimal after the proposed reallocation algorithm as shown in Table 8.

**Step 4 .**

implementation of the spiral technique as mentioned in the previous section. Generate a bubble plan (Figure 5) and thus the resulting modified initial layout plan Figure 6 as shown in Table 9.

**Step 5 .**

Using

(3) $$\begin{array}{c} {LS}^{a}=\overset{M-1}{\underset{i=1}{\sum }}\overset{M}{\underset{j=j+1}{\sum }}V\left(r_{ij}\right).a_{ij}\text{.} \end{array}$$

Layout score after reallocation = 41.5.

The resulting layout score of the proposed design is 41.5. This score was raised by 32.5%, leading to the enhanced OT layout design as shown in Figure 6.

Therefore, the redesign process according to the proposed algorithm in this selected case is optimal to enhance the status of the selected department in the selected hospital to meet the international standards for healthcare facilities.

And so on for the other operating theater at the selected hospitals, as shown in Figure 7.

### 4.2. Emergency Department Reallocation Case Study

The reallocation process of the Emergency Departments showed that the layout score before applying the proposed algorithm for reallocation is 18%. The ED at hospital I is shown in Figure 8.

**Step 6 .**

extracted REL chart as shown in Table 10 for the Emergency Department in hospital I.

**Step 7 .**

extracted adjacency matrix from the proposed adjacency matrix as shown in Table 11 for the Emergency Department in hospital I.

**Step 8 .**

adjacency matrix for the Emergency Department as optimal after the proposed reallocation algorithm as shown in Table 12.

**Step 9 .**

implementation of the spiral technique, as mentioned in the previous section. Generate a bubble plan (Figure9) and thus the resulting modified initial layout plan (Figure 10) as shown in Table 12.

And so on for any healthcare departments, as shown in Figure 11.

## 5. Conclusion

Measuring service quality is one of the most important challenges of our time. In this kind of investigation, the client's perceptions about services must be analyzed, and the services should be designed according to the results of the investigations. In picking up the problems of the best-performing hospital, various alternatives were envisaged and assessed according to a number of criteria.

This study offers a scientific way to evaluate hospital decision. The triangular fuzzy numbers were used to express the linguistic variables collected from surveys. The MCDM approach was used for synthesizing the decision. Determining and ranking the overall performance values of the hospital departments was managed with the TOPSIS method. In this particular study, the topic in question is to determine the benefits of the redesign decision of hospital departments to meet international standards. Hospital D indicates the highest rank performance in all departments. Hospital I receives the lowest rank in most of its departments.

This ranking algorithm helps the decision-makers make the optimal decision for any procedure required to enhance healthcare services.

Reallocation of the department Operating theater spaces in hospital F in the ranked evaluated hospitals was carried out by a graph theoretic heuristic. The adjacency matrix was used to reflect the closeness rating of the spaces in the operating theater. A manual qualitative technique called the spiral technique was used to derive the initial layout block plan. Satisfactory results were obtained. Operating theater layout designs were improved by up to 32.5%. This lets to make a decision for redesigning the selected departments in the selected hospital.

We will apply the proposed methodology to more healthcare facilities and present the improvement after redesigning these facilities as future work and applying ranking new methods compared with the TOPSIS technique.

## Figures and Tables

**Figure 1:** Linguistic scales for the rating of each department.

**Figure 2:** Proposed ranking model.

**Figure 3:** Flowchart of the proposed decision-making algorithm.

**Figure 4:** Case study: operating theatre plan.

**Figure 5:** Bubble plan operating theater in hospital F after reallocation.

**Figure 6:** Layout plan of the operating theater department after applying the reallocation proposed algorithm.

**Figure 7:** Layout score after and before applying the reallocation proposed algorithm and the enhancement percentage for the operating theatre in the selected hospitals.

**Figure 8:** Case study: Emergency Department in hospital I plan.

**Figure 9:** Bubble plan Emergency Department in hospital I after reallocation.

**Figure 10:** Layout plan of the Emergency Department in hospital (I) after applying the reallocation proposed algorithm.

**Figure 11:** Layout score after and before applying the reallocation proposed algorithm and the enhancement percentage for the Emergency Department of the selected hospitals.

**Algorithm 1:** Hospitals' departments evaluated: ranking using the fuzzy TOPSIS method.

**Algorithm 2:** Reallocation of department's area.

**Table 1:** Summary of the studies that used ranking methods.

Study	Used algorithms								
	TOPSIS	MOORA	VIKOR	PROMETHEE	SAW	COMET	CODAS	SIMUS	CODAS-COMET
Assessment of service quality in teaching hospitals of Yazd university of medical sciences: using multicriteria decision-making techniques [8]	Yes	No	No	No	No	No	No	No	No
A healthcare facility location selection problem with fuzzy TOPSIS method for a regional hospital [9]	Yes	No	No	No	No	No	No	No	No
Assessment of performance in teaching hospitals: using multicriteria decision-making techniques [10]	Yes	No	No	No	No	No	No	No	No
Beheshtinia. Evaluating and prioritizing hospital service quality [11]	Yes	No	No	No	No	No	No	No	No
Determination of hospital rank by using the technique for order preference by similiarity to ideal solution (TOPSIS) and multiobjective optimization on the basis of ratio analysis (MOORA) [12]	Yes	Yes	No	No	No	No	No	No	No
Multiobjective contractor's ranking by applying the MOORA method [13]	No	Yes	No	No	No	No	No	No	No
Determination of hospital rank by using analytic hierarchy process (AHP) and multiobjective optimization on the basis of ratio analysis (MOORA) [14]	No	Yes	No	No	No	No	No	No	No
Hospital leanness assessment model: a fuzzy MULTI-MOORA decision-making approach [15]	No	Yes	No	No	No	No	No	No	No
Measuring the quality of public hospitals in Croatia using a multicriteria approach [16]	No	Yes	No	No	No	No	No	No	No
Identifying and ranking health tourism development barriers in Iran using the fuzzy VIKOR method [17]	No	No	Yes	No	No	No	No	No	No
Implications for sustainable healthcare operations in embracing telemedicine services during a pandemic [18]	No	No	Yes	No	No	No	No	No	No
Bastani. Ranking of Iranian provinces based on healthcare infrastructures: Before and after implementation of health transformation plan [19]	No	No	Yes	No	No	No	No	No	No
PROMETHEE-based analysis of HCWM challenges in the healthcare sector of Odisha [20]	No	No	No	Yes	No	No	No	No	No
Improving decision-making and management of hospital resources: an application of the PROMETHEE II method in an emergency department [21]	No	No	No	Yes	No	No	No	No	No
Stability of hospital rankings [22]	No	No	No	Yes	No	No	No	No	No
Ranking of hospitals in the case of COVID-19 outbreak: a new integrated approach using patient satisfaction criteria [23]	No	No	No	No	Yes	No	No	No	No
The COMET method: the first MCDA method completely resistant to rank reversal paradox [24]	No	No	No	No	No	Yes	No	No	No
The COMET rating procedure in practice: some conclusions [25]	No	No	No	No	No	Yes	No	No	No
Effects of the selection of characteristic values on the accuracy of results in the COMET method [26]	No	No	No	No	No	Yes	No	No	No
A novel fuzzy SIMUS multicriteria decision-making method. An application in railway passenger transport planning [27]	No	No	No	No	No	No	Yes	No	No
A new combinative distance-based assessment (CODAS) method for multicriteria decision-making [28]	No	No	No	No	No	No	No	Yes	No
Green electricity generation assessment using the CODAS-COMET method [29]	No	No	No	No	No	No	No	No	Yes

**Table 2:** Summary of ranking methods: benefits and limitations [32].

Methods	Benefits	Limitations
TOPSIS	Provides the option of the most excellent stable performance results when input information changes Informal in terms of maintaining similar steps regarding the size of the problem Extensively used for several areas, such as logistics, engineering, and environmental management Permits to deduce the absolute estimation of a particular alternative Is based on a modest process and is easy to apply and programmable	It is not easy to weigh and keep the consistency of judgment, particularly with added attributes The submission of Euclidean space does not look at the connection between the attributes
MOORA	More vital than others and involve all related investors interested in specific issues such as an advantage Grounded on quantitative numbers and stronger than others based on ordinal processes Nonsubjective on one side and more vital in linking with methods using subjective estimations to implement the selection for objective significance	This method has one major disadvantage in the information of objectives applied in the database when data cannot be the same as zero or deal with negative figures
VIKOR	Used in defining the steadiness intervals in weights Supports multicriteria decision-making (MCDM) when an individual has no idea to express one's preference Based on the principle of MCDM systems cooperation programming The cooperation solution in this method will be changed if the measure of weight does not suit the stability interval Requires normalization	Require initials weights Suitable in such cases when data are arithmetical values The ranking requirement can be performed with the changed value of variable weights
PROMETHEE	Easy to apply Does not need the criteria to be equivalent Requires normalization Not required to reduce the variable and the information transformation if this approach is not inaccurate	Does not provide a transparent background for assigning the weights Requires the assignment of measures but does not provide an understandable background to assign the values
SAW	Can compensate in the middle of the variables Participates in the value of variables and weights into a particular one greatness Is appropriate to appraise a single alternative The calculation process is not complex and can be executed without a computer system Regularized values of the appraisal assist in visually calculating the changes between the alternatives	Is grounded on normalization by reducing the variables and changing to maximizing Estimates generated do not always reflect the actual status. The answer might not be in terms of logic The primary dimension of the variable is possibly about unity, whereas the most nominal size might reach zero Might be applied if every variable is maximized before breakdown

**Table 3:** Fuzzy sets for evaluation choices.

Linguistic variables	Corresponding triangular fuzzy numbers
Satisfied	(0.0, 0.2, 0.4)
Can be satisfied	(0.2, 0.4, 0.6)
Not applicable	(0.6, 0.8, 1)

**Table 4:** Hospital characteristics.

Hospital	No. departments	Size (no. beds)
A	13	402
B	11	87
C	11	83
D	14	301
E	11	63
F	11	214
G	13	274
H	13	180
I	13	340
J	12	210

**Table 5:** Survey's structure: standards and criteria.

Standards	Criteria	Subcriteria
AIA (American Institution of Architecture) [41]	Guidelines for design and construction of healthcare facilities	Spaces, finishing, doors, and windows design
FGI (Facility Guideline Institution) [41]	Guidelines for design and construction of healthcare facilities	Spaces, finishing, doors, and windows design
JCAHO (Joint Commission on Accreditation of Healthcare Organizations) [42]	Planning, design, construction of healthcare facilities	Spaces, finishing, doors, and windows design
ICRA (Infection Control Risk Assessment) [43]	Focuses on risk reduction from infection, acts through phases of facility planning, design, construction, renovation, facility maintenance, and coordinates and weighs knowledge about infection, infectious agents, and care environment, permitting the organization to anticipate the potential impact	Number, location, and type of airborne infection isolation and protective environment rooms, location of special ventilation and filtration, such as emergency department waiting and intake areas., air handling, and ventilation needs in surgical services, airborne infection isolation and protective environment rooms, laboratories, local exhaust systems for hazardous agents, and other special areas, water systems to limit *Legionella* sp. And other waterborne opportunistic pathogens, finishes, and surfaces
ASHRAE (American Society of Heating, Refrigerating, and Air-conditioning Engineering) [42]	Heating, ventilation, air conditioning, and refrigeration systems design and construction	Heating, ventilation, air conditioning, and refrigeration criteria
HTM 2022 (Health Technical Memorandum) [44, 45]	Covers piped medical gases, medical compressed air, and medical vacuum installations and apply to all medical gas pipeline systems installed on healthcare premises	Medical gases distribution, piping distribution criteria

**Table 6:** Evaluated hospitals: department ranking.

Hospitals	Pediatric critical care unit	CCU	NICU	CCCU	Radiology	Nurseries	OR	Nuclear medicine	Emergency	Laboratory	Hemodialysis	Gastrointestinal endoscopy	Nursing units	Cardiac catheterization laboratory
A	4	4	4	5	3	2	3	—	4	2	2	2	3	3
B	5	5	7	9	7	5	9	—	10	5	9	—	6	—
C	6	7	10	10	9	3	10	—	9	7	7	—	7	—
D	1	1	1	1	1	1	1	1	1	1	1	1	1	1
E	7	6	5	7	10	8	7	—	8	10	5	—	8	—
F	9	3	9	2	4	4	8	2	5	4	4	3	2	2
G	8	10	2	3	2	6	2	3	3	3	3	7	9	—
H	2	2	8	4	5	9	4	—	2	9	8	4	5	4
I	10	8	6	6	8	10	6	4	7	8	6	6	10	—
J	3	9	3	8	6	7	5	—	6	6	10	5	4	—

**Table 7:** Proposed adjacency matrix (present).

No	Area	4	7	12	14	18	23	24	25	26
4	Staff clothing change areas		0.5	1	0	0	0.5	0.5	0	0
7	Semirestricted corridor			0.5	0.5	0.5	1	0.5	0.5	0.5
12	Offices				0	0	0	0	0	0
14	Report preparation area					0	0.5	0	0.5	0
18	Medicine dispensing unit						0	0.5	0.5	0
23	Operating and procedure rooms							1	0.5	0.5
24	Clean core								0.5	0.5
25	Scrub sink areas									0
26	A substerile service area									

**Table 8:** Extracted REL chart for the operating theater department.

No	Area	4	7	12	14	18	23	24	25	26
4	Staff clothing change areas		E	O	O	U	O	E	I	U
7	Semirestricted corridor			O	O	A	U	A	O	O
12	Offices				E	U	U	U	U	U
14	Report preparation area					U	U	U	U	U
18	Medicine dispensing unit						I	I	U	U
23	Operating and procedure rooms							A	E	E
24	Clean core								A	A
25	Scrub sink areas									E
26	A substerile service area									

**Table 9:** Extracted adjacency matrix for the operating theater department after the reallocation process.

No	Area	4	7	12	14	18	23	24	25	26	TCR	Order
4	Staff clothing change areas	0	1	0	0	0	0	0.5	0	0	1.5	8
7	Semirestricted corridor	0	0	1	1	1	0	1	0	0	4	2
12	Offices	0	1	0	1	0	0	0	0	0	2	5
14	Report preparation area	0	1	1	0	0	0	0	0	0	2	6
18	Medicine dispensing unit	0	1	0	0	0	0	0	0	0	1	9
23	Operating and procedure rooms	0	0	0	0	0	0	1	1	1	3	3
24	Clean core	0.5	1	0	0	0	1	0	1	1	4.5	1
25	Scrub sink areas	0	0	0	0	0	1	1	0	0	2	7
26	A substerile service area	0	0	0	0	0	1	1	1	0	3	4

**Table 10:** Emergency Department REL matrix in selected hospital [it is reproduced from [39] in the mentioned format under a creative commons attribution 4.0 international license].

	Area	1	2	3	4	5	6	7	8	9	10	11
1	Entrance		A	U	A	A	O	A	O	O	O	O
2	Equipment and supply storage			A	O	O	O	O	O	O	O	O
3	Staff lounge				O	E	O	O	O	O	O	O
4	Public waiting area					A	U	E	I	I	I	I
5	Diagnostic service areas						X	I	E	I	E	I
6	Patient toilet							A	I	O	O	O
7	Shower room								A	O	E	I
8	Airborne infection isolation (AII) room									U	A	E
9	Multiple-bed treatment room (s)										U	A
10	Reception, triage, and control station											U
11	A trauma/resuscitation room (s)											

**Table 11:** Emergency Department adjacency matrix in selected hospital (I) [it is reproduced from [39] in the format under a creative commons attribution 4.0 international license].

	Area	1	2	3	4	5	6	7	8	9	10	11
1	Entrance		0	0	0.5	0	0	0	0	1	1	0
2	Equipment and supply storage			0	0	1	0	0	0	0	0	0
3	Staff lounge				0.5	0.5	0	0	0	0	0	0
4	Public waiting area					0.5	0.5	0.5	0.5	0.5	0.5	0.5
5	Diagnostic service areas						0	0	0	0	0	0
6	Patient toilet							1	0.5	0	0	0
7	Shower room								1	0	0	0
8	Airborne infection isolation (AII) room									0	0	0
9	Multiple-bed treatment room (s)										0.5	0.5
10	Reception, triage, and control station											1
11	A trauma/resuscitation room (s)											

**Table 12:** Extracted adjacency matrix for the Emergency Department at hospital (I) after the reallocation process.

	Area	1	2	3	4	5	6	7	8	9	10	11	TCR	Order
1	Entrance	0	0	0	2	0	0	0	0	1	1	0	4	3
2	Equipment and supply storage	0	0	0	0	1	0	0	0	0	0	0	1	6
3	Staff lounge	0	0	0	0.5	1.5	0	0	0	0	0	0	2	4
4	Public waiting area	0	0	0	0	2	0	1.5	1	1	1	1	7.5	1
5	Diagnostic service areas	0	0	0	0	0	0	0	0	0	0	0	0	7
6	Patient toilet	0	0	0	0	0	0	4	1	0	0	0	5	2
7	Shower room	0	0	0	0	0	0	0	0	0	0	0	0	8
8	Airborne infection isolation (AII) room	0	0	0	0	0	0	0	0	0	0	0	0	9
9	Multiple-bed treatment room (s)	0	0	0	0	0	0	0	0	0	0	2	2	5
10	Reception, triage, and control station	0	0	0	0	0	0	0	0	0	0	0	0	10
11	A trauma/resuscitation room (s)	0	0	0	0	0	0	0	0	0	0	0	0	11

Layout score before applying the reallocation proposed algorithm = 18. Layout score after applying reallocation proposed algorithm = 24.75 that raised by 27%. and so on for every emergency department in the evaluated hospitals.

## Data Availability

The data supporting this study's findings are available from the corresponding author upon reasonable request.
